The article "Chimeric antigen receptors: unleashing a new age of anti-cancer therapy" was published in 2018. Journal: Cancer Cell Int.

# Chimeric antigen receptors: unleashing a new age of anti-cancer therapy

**DOI:** 10.1186/s12935-018-0685-x

**Published:** 2018-11-14

**Authors:** Yan Leyfman

**Affiliations:** Penn State College of Medicine, 61A University Manor East, Hershey, PA USA

**Keywords:** Chimeric antigen receptor, Leukemia, Hematological malignancy, T cell, Immunotherapy, Solid tumor, CAR resistance

## Abstract

**Background:**

Chimeric antigen receptors (CARs) represent a novel facet of modern day synthetic biology that exemplifies personalized medicine at work through their ability to harness and redirect a patient’s immune system to fight cancer.

**Body:**

By combining the target-specificity of antibodies to the effector capabilities of T cells, CARs have yielded high remission rates for many late staged and relapsed/refractory (r/r) hematological malignancies, including acute lymphoblastic leukemias (ALL) and Non-Hodgkin’s lymphomas. Despite toxicities of cytokine release syndrome and neurotoxicity, recent studies have uncovered their underlying mechanisms and devised effective therapies to manage and possibly prevent them. In 2017, CAR T cell therapy became a reality for the general public despite the high costs, when Novartis’s Kymriah, became the first product to receive FDA approval for pediatric r/r B cell ALL with Gilead’s Yescarta following several months later. Although effective in hematological malignancies, CAR response has been limited in solid tumors largely attributed to the heterogeneous and immunosuppressive tumor microenvironment along tumor defense mechanisms, such as antigenic escape.

**Conclusion:**

Despite the current challenges of CAR T therapy, this technology is still in its infancy and its promise will continue to grow as scientists continue to develop novel approaches to enhance its efficacy. As its prevalence continues to increase, institutions and pharmaceuticals worldwide are investing in this technology in hopes of driving therapeutic innovation, while providing greater access to their respective populations through clinical trials.

## Introduction and history

Since 1935, cancer has remained the second leading cause of death in the United States with a steadily increasing number of new cases yearly [1]. Although standard anti-cancer drugs, which are predominantly nonselective cellular poisons that indiscriminately target the most metabolically active cells, are used, cancer mortality rates remained constant from 1950 to 2005 in late stage disease according to the American Cancer Society [2]. Medication prices, however, have continued to skyrocket with increases by as much as 1400% since 1976 for certain cancer subtypes [1]. Scientists believed that they could rectify this by harnessing the power of a patient’s immune system to fight this disease; this in turn led to the development of CAR T cell therapy—an example of personalized medicine at work, whereby each patient’s immune cells can act as a living drug to enhance the immune response to combat disease.

Chimeric antigen receptor T cells, a unique facet of modern-day synthetic biology, combine the targeted specificity of antigens with the downstream intracellular signaling potential of a T cell receptor to enhance T cell potency and function [3]. Interaction with antigen leads to CAR activation and the turning on of downstream T cell signaling pathways to yield cytotoxic killing through granzymes and perforins and enhanced immune response through cytokine release [4]. First-generation CARs, which consisted of only an HLA-independent extracellular domain and an intracellular T cell activating domain comprised of the zeta chain of the CD3 complex, exhibited limited efficacy due to their inability to sustain T cell signaling responses [5]. This was rectified with the creation of second-generation CARs, which contained a co-stimulatory receptor to enhance T cell function, expansion, and efficacy [6]. Third generation CARs have multiple co-stimulatory domains to further enhance T cell function and efficacy [3]. Achieving successful results at the bench, second-generation CARs entered clinical trials in 2009. In this single treatment, a patient’s T cells were harvested, activated ex vivo with antibody-coated beads, transduced with a lentiviral vector bearing the CAR, expanded, purified, cryopreserved, assessed for quality, and then reinfused into the patient after conditional chemotherapy (Fig. 1) [7]. The quality control assessment is based on the United States Food and Drug Administration (USFDA) protocol guidelines that assesses safety, sterility and potency. Safety testing is performed to show that this product can be given to humans without harm. Sterility testing ensures that the product is without microbiological contaminants and free from impurities, including remnants of assays, vectors, and growth media. Vector product potency is performed to ensure that the identity and function of the CAR product are what it should be [8]. Direct clinical application of this protocol was first performed in 2010 by physicians at the National Cancer Institute who were the first to demonstrate the clinical efficacy of CAR T cell therapy, when they successfully induced regression of advanced lymphoma in one patient [9]. In 2011, Memorial Sloan Kettering Cancer Center (MSKCC) became the first institution to demonstrate complete remission of relapsed/refractory B-cell acute lymphoblastic leukemia (r/r B-ALL) in 8 patients in their Phase I clinical trial [10]. When expanded to 38 patients, the overall complete remission rate in this trial was 87% with a median time to complete remission lasting only 23 days and a complete bone marrow recovery within 2 months [11]. In 2012, similar results for r/r B-ALL were demonstrated by the Children’s Hospital of the University of Pennsylvania when 7-year old Emily Whitehead successfully achieved complete remission [12].

**Fig. 1:** CAR T Cell Manufacturing Process. Initially, leukophoresis is performed to separate out the patient’s immune cells from the rest of the patient’s constituents of blood. Isolated T lymphocytes are enriched through counterflow, which separates cells by size and density to maintain their viability. Next, beads containing anti-CD3/antiCD-28 antibodies are added to activate the T cells. During the activation process, the T cells are incubated with a CAR-encoding lentiviral vector, which integrates the CAR into the T cell through reverse transcription. T cell expansion is performed within a bioreactor for 9–11 days, after which time the magnet beads are removed from culture. Subsequently, CAR T cells are washed, concentrated, and cryopreserved at − 80 °C. Quality control checks for safety, sterility, and vector potency are performed per USFDA protocol guidelines. The patient is given conditional chemotherapy, T cells are re-infused, and the patient is monitored for any adverse reactions for a period of 7–10 days [8]

## Side effects and solutions

Despite these clinical successes, CAR T cells have been shown to cause several potent side effects. Cytokine release syndrome (CRS) occurs when CARs overstimulate the immune response through cytokine release leading to respiratory distress, hypotension and fever [10]. Physicians are able to adequately control this with Tocilizumab (a humanized monoclonal antibody against the IL-6 receptor) and high dose steroids if refractory [11]. However earlier this year, scientists discovered that CRS is actually caused by macrophages hypersecreting IL-1 and can be effectively managed by IL-1 receptor inhibitors, such as Anakinra [13].

Another potent side effect of this therapy is neurotoxicity, which can have a diverse clinical presentation ranging from delirium and aphasia to global encephalopathy and seizures [11]. Although the root cause of these toxicities is uncertain, several studies have suggested that they may arise from semi-random mutagenesis when using a retroviral vector during the transduction phase of CAR T cell manufacturing, as viruses have the potential of integrating randomly within the genome including near oncogenic sites [14, 15]. Although CAR T cell viral vector-mediated oncogenicity has not been directly observed, it is still a concern of the FDA, which recommends follow-up for up to 15 years to monitor adverse effects [16, 17]. To rectify this, scientists from MSKCC used a gene targeting platform of CRISPR/CAS9, *in lieu* of viruses, to directly target the T-cell receptor α constant (TRAC) locus during the transduction phase of CAR T cell development minimizing off-target effects. This approach resulted in more uniform CAR expression with enhanced T cell potency in an ALL mouse model with minimal side effects [18]. These positive results suggest that modifications in CAR T cell manufacturing can have a profound impact and yield more effective CARs with reduced side effects.

## CAR products on the market

The potential of CAR T cells therapy was realized in August 2017 when Novartis’s second-generation CD19-targeted CAR T product containing a 4-1BB-derived costimulatory domain, Kymriah, became the first treatment to receive FDA approval for pediatric r/r B-cell ALL. Several months later, Gilead’s Yescarta (formerly known as Kite Pharma) received FDA approval for the treatment of Diffuse Large B cell lymphoma [19]. Yescarata, although a CD19-targeted CAR just like Kymriah, contains a CD28 co-stimulatory domain [20]. Celgene’s Liso-cel (formerly known as Juno Therapeutics), indicated for Diffuse Large B cell, Non-Hodgkin’s, follicular, mantle cell, and primary mediastinal B cell lymphomas, will be submitted for FDA approval before the end of 2018 [19]. Although it is structurally similar to the product from Novartis’s with a 4-1BB costimulatory domain, the product utilizes a different manufacturing cell composition consisting of both CD4 and CD8 T cells compared to the others which only use CD4. Over a 6-month period, Liso-cel, in a cohort of 67 patients, demonstrated a 50% complete remission where only 1% of patients developed severe CRS and 15% experienced severe neurotoxicity, while Yescarta showed a 36% complete remission in 101 patients where 13% developed CRS and 31% experienced severe neurotoxicity [21]. In a cohort of 81 patients, Kymriah showed a 30% complete response with only 23% experiencing CRS and 12% severe neurotoxicity [21].

Despite their efficacy, the cost of therapy will become a major concern with Kymriah costing $475,000 per infusion, while Yescarta will be priced at $373,000 [22]. However, manufacturers have a adopted a model of value-based pricing where patients only pay if they respond by the first month post-infusion [22]. In the United States, the Centers for Medicare & Medicaid Services will compensate Novartis $500,839 and Gilead $395,380, respectively, for their therapies administered in the out-patient setting and have set a maximum patient out-of-pocket expense of $1340 as of 2018 [23]. Although most insurances cover this therapy, manufacturers have devised grants to help those unable to afford treatment. Irrespective, future accessibility of this therapy will largely hinge on affordability as this will determine the number of centers that can offer this treatment to their patients.

## CAR T cell resistance and application to solid tumors

Although CAR T cells have transformed the treatment of patients with r/r B-ALL, several patients have experienced relapse post-therapy [24]. Although the sample is small, studies from patients have shown antigen escape, where relapsed patients with the same malignancy lack express of CD19 rendering CAR targeting ineffective [25]. A potential solution could be to target multiple antigens on cancer cells through engineering either multi-antigen CAR T cells or utilizing multiple CARs each targeting a different antigen [26]. However such an approach may be limited by additional costs of CAR T cell development. Certain hematological malignancies, such as lymphomas, have demonstrated an increased expression of inhibitory ligands, such as SHP-1 PD-1, CTLA-4, TIM-3, LAG-3 and A2AR [27]. To combat this, scientists have proposed combining CAR T cells with checkpoint inhibitors, which have demonstrated improved efficacy in mice [27]. Early clinical trials from B-ALL pediatric patients treated with pembrolizumab (humanized anti-PD-1 antibody) and CD-19-specific CAR T cells showed improved clinical responses and prolonged CAR T cell persistence [28]. Additionally, a recent study has noted the presence of transduction-induced CAR T cell resistance in a relapsed B-ALL patient post therapy, where leukemic cells were found to be transduced with the CAR protein in addition to the T cell [29]. This allowed the leukemic cell to evade initial CAR therapy and ultimately promote disease relapse. Thus, this illustrates the importance of clean CAR T cell manufacturing to minimize unwanted therapeutic complications.

Despite instances of CAR resistance in hematological malignancies, CAR efficacy in solid tumors has been severely limited. Studies have attributed this to a heterogenous tumor microenvironment that minimizes the number of specific cell surface tumor antigens along with a microenvironment that limits CAR trafficking due to chemokine receptor mismatch, expression of immunosuppressive agents like prostaglandin E2 and cyclooxygenase 2, and presents an unfavorable metabolic environment that severely limits CAR efficacy [30]. Just like their r/r hematological counterparts, solid tumors have also been shown to exhibit antigenic escape [30]. To circumvent this, researchers at the University of Pennsylvania have proposed designing CARs targeting the unique molecular signatures of cancer cells exhibited in their *O*-linked glycosylation sites, while researchers at MSKCC have designed secretable CARs, called “Armored CARs” [31–33]. This new iteration of CAR T cells expresses a co-stimulatory molecule with a secretable IL-12 cytokine that enhances chemotaxis to solid tumors, provides greater immunological persistence, decreases cellular exhaustion, and affords enhanced cytotoxicity with resistance to the inhibitory tumor microenvironment [33]. Recent animal studies against ovarian cancer utilizing MUC-1616-targeted Armored CAR T cells co-expressing PD-1 checkpoint inhibiting antibodies have been shown to possess more efficacious anti-tumor responses, longer CAR persistence, and enhanced T cell activation contributing to improved mouse longevity [34]. Thus, this indicates that future CAR enhancements can aid in circumventing the resistant tumor microenvironment to attain better disease control and ultimately result in improve patient mortality.

## Novel developments and current clinical trials

To circumvent the challenges and present limitations of CAR T cell monotherapy, scientists have suggested the use of combinational therapies to enhance CAR efficacy. For instance, several recent studies have shown that combining chemotherapy with CAR T cells can reduce disease burden, improve tumor antigen recognition, and enhance CAR T cell efficacy and persistence [35–38]. Other studies have suggested that radiotherapy can serve to enhance CAR T cell efficacy by sensitizing tumor cells to cytotoxic lymphocytes, enhance the trafficking and infiltration of T cells, improve antigen presentation on tumor cells, and promote overall T cell survival [39–43]. To combat the immunosuppressive microenvironment induced particularly by solid tumors, studies have augmented CAR T cell therapy with checkpoint inhibitors, such as anti-PD-1 (nivolumab, pidilizumab and pembrolizumab), anti-PD-L1 (MDX-1105), and anti-CTLA-4 (ipilimumab), and have demonstrated improved tumor regression, increased long-term survival in mice and have improved CAR efficacy and persistence in clinical trials [44, 45]. It is hoped that these approaches will serve to enhance the effectiveness of CAR T cell therapy and promote a more potent anti-cancer response. Nonetheless, this technology has already demonstrated its merit through its ability to induce complete remission in certain late stage cancers. As this technology continued to be refined, its prevalence will only continue to grow as evident by the increasing number of CAR T cell clinical trials. For instance, over 200 clinical trials against malignancies such as glioblastomas, neuroblastomas, prostate, pancreatic, lung, liver and breast cancers have opened up within the past year worldwide [46]. Although time will tell whether CAR T cell therapy will 1 day circumvent standard therapies of care for certain oncological malignancies, medicine has a new weapon of precision in the longstanding battle with cancer.

## Abbreviations

ALL: acute lymphoblastic leukemia
CAR: chimeric antigen receptor
CRS: cytokine release syndrome
MSKCC: Memorial Sloan Kettering Cancer Center
r/r: relapsed/refractory
TRAC: T-cell receptor α constant
USFDA: United States Food and Drug Administration
